# Symptom-Based COVID-19 Prognosis through AI-Based IoT: A Bioinformatics Approach

**DOI:** 10.1155/2022/3113119

**Published:** 2022-07-23

**Authors:** Madhumita Pal, Smita Parija, Ranjan K. Mohapatra, Snehasish Mishra, Ali A. Rabaan, Abbas Al Mutair, Saad Alhumaid, Jaffar A. Al-Tawfiq, Kuldeep Dhama

**Affiliations:** ^1^Electronics and Communication Engineering, CV Raman Global University, Bidyanagar, Mahura, Janla, Bhubaneswar, Odisha 752054, India; ^2^Department of Chemistry, Government College of Engineering, Keonjhar, Odisha 758002, India; ^3^Bioenergy Lab, School of Biotechnology, Campus-11, KIIT Deemed University, Bhubaneswar, Odisha 751024, India; ^4^Molecular Diagnostic Laboratory, Johns Hopkins Aramco Healthcare, Dhahran 31311, Saudi Arabia; ^5^College of Medicine, Alfaisal University, Riyadh 11533, Saudi Arabia; ^6^Department of Public Health and Nutrition, The University of Haripur, Haripur 22610, Pakistan; ^7^Research Center, Almoosa Specialist Hospital, Al-Ahsa 36342, Saudi Arabia; ^8^College of Nursing, Princess Norah Bint Abdulrahman University, Riyadh 11564, Saudi Arabia; ^9^School of Nursing, Wollongong University, Wollongong NSW 2522, Australia; ^10^Administration of Pharmaceutical Care, Al-Ahsa Health Cluster, Ministry of Health, Al-Ahsa 31982, Saudi Arabia; ^11^Specialty Internal Medicine and Quality Department, Johns Hopkins Aramco Healthcare, Dhahran 31311, Saudi Arabia; ^12^Indiana University School of Medicine, Indiana 46202, USA; ^13^School of Medicine, Johns Hopkins University Baltimore, MD 21287, USA; ^14^Division of Pathology, ICAR-Indian Veterinary Research Institute, Izatnagar, Bareilly, 243122 Uttar Pradesh, India

## Abstract

**Objective:**

Internet of Things (IoT) integrates several technologies where devices learn from the experience of each other thereby reducing human-intervened likely errors. Modern technologies like IoT and machine learning enable the conventional to patient-specific approach transition in healthcare. In conventional approach, the biggest challenge faced by healthcare professionals is to predict a disease by observing the symptoms, monitoring the remote area patient, and also attending to the patient all the time after being hospitalised. IoT provides real-time data, makes decision-making smarter, and provides far superior analytics, and all these to help improve the quality of healthcare. The main objective of the work was to create an IoT-based automated system using machine learning models for symptom-based COVID-19 prognosis.

**Methods:**

Comparative analysis of predictive microbiology of COVID-19 from case symptoms using various machine learning classifiers like logistics regression, k-nearest neighbor, support vector machine, random forest, decision trees, Naïve Bayes, and gradient booster is reported here. For the sake of the validation and verification of the models, performance of each model based on the retrieved cloud-stored data was measured for accuracy.

**Results:**

From the accuracy plot, it was concluded that k-NN was more accurate (97.97%) followed by decision tree (97.79), support vector machine (97.42), logistics regression (96.50), random forest (90.66), gradient boosting classifier (87.77), and Naïve Bayes (73.50) in COVID-19 prognosis.

**Conclusion:**

The paper presents a health monitoring IoT framework having high clinical significance in real-time and remote healthcare monitoring. The findings reported here and the lessons learnt shall enable the healthcare system worldwide to counter not only this ongoing COVID but many other such global pandemics the humanity may suffer from time to come.

## 1. Introduction

The ongoing COVID-19 pandemic is caused by a highly contagious novel virus, namely, severe acute respiratory syndrome coronavirus 2 (SARS-CoV-2). After its official report of origin from Wuhan, China, on 31 December 2019, the pathogen spread astoundingly fast round the globe and emerged as a global pandemic [1–3]. As this report is being drafted (7 July 2021), more than 3.9 million global tally of deaths is registered attributed mainly to the human-to-human viral transmission [4]. This novel and rapidly evolving mutating RNA virus has not only attacked the health and medical systems but also the global economy significantly, rewriting socioeconomic activities including the stock and financial markets [1, 2]. It has also affected the cultural, social, festival, and knowledge-sharing activities and the overall human behavioural patterns [1]. The human-to-human transmission mainly occurs through respiratory droplets/aerosols and the faecal-oral route [5]. Several other means of transmissions include air-borne transmission and direct/indirect contacts (such as the fomite) [6]. The disease is manifested with typical [5, 7] and atypical [8, 9] symptoms. As per reports, the virus infects the upper and lower respiratory parts, heart, kidney, liver, gut, and the nervous system, ultimately causing multiorgan damage [10, 11]. It causes severe health problems in the immunocompromised with diabetes, obesity, hypertension, cardiovascular disorder, psychiatric disorder, etc. [12–14].

Numerous measures have been taken by the health bodies and the government agencies to combat SARS-CoV-2 transmission. Since the onset of the novel virus, healthcare professionals have gone that extra mile to help the needy. A major challenge faced by them is the shortage of testing kits and other medical equipment. As a result, the pandemic continues to challenge the medical systems all around [15]. In such a scenario, an early diagnosis of the disease may improve the healthcare facility. This research article focuses on predictive COVID-19 prognosis using machine learning (ML) algorithm. Machine learning is a subset of artificial intelligence (AI) that uses statistics to enable machines to improve with experience.

ML algorithm categorises into three types, supervised (task driven), unsupervised (clustering), and reinforcement learning. Supervised learning algorithm handles two types of problems, classification and regression. Learning algorithm takes samples as input (training set). Unsupervised learning algorithm predisposes unlabelling for unbiased prediction. In reinforcement learning (RL), the agent learns to interact with the environment to achieve a reward. It has promising application for rational decision making in diverse fields, such as energy management, robotics, agriculture, and healthcare. Moreover, Kumar et al. have developed the deep learning and reinforcement learning models to forecast COVID-19-infected individuals, losses, and cures with the predictive outcomes [16]. Wang et al. have also applied the reinforcement learning method to detect COVID-19 infection [17]. In the real-time monitoring platform based on IoT devices, Fang et al. [18] focused on energy harvesting in next-generation multiple access systems with the objective of data sensing and transmission using different multiple access networks. The study draws substantial attention to the low peak age of information (AoI) at low power consumption. Abd-Elmagid et al. [19] have described the comparison among delay, throughput, and age of information. The study explored the optimal sampling policy that combines wireless energy transfer with the objective of minimizing long-term weighted sum-AoI.

Under the current study, the authors have endeavoured to apply different ML techniques and publicly available cloud-stored healthcare datasets to build a system that allows real-time and remote health monitoring built on IoT and is associated with cloud computing. Such system shall be allowed to derive recommendations based on the past and empirical data stored in the cloud. IoT is a progressive technology that is drastically evolving and improving day by day with advancements in information technology and allied technologies. The main objective of the study was applying ML models to predict COVID-19 by observing the symptoms manifested by the patients using the real-time data. Applying ML in predicting COVID-19 infection adds a new dimension to early disease diagnosis. It would help researchers as well the medical professionals in predicting the rising cases of COVID-19 from symptoms and also help prevent the pandemic with due precaution and prevention.

Recently, Pourhomayoun and Shakibi [20] proposed a model that integrated AI and machine learning to forecast the mortality rate in COVID-19 cases. They analysed the data of more than 2,670,000 samples of confirmed COVID cases from 146 countries and reported 89.98% prediction accuracy in the mortality rate COVID-19 patients [20]. Muhammad et al. [21] compared five supervised machine learning models, LR, DT, SVM, NB, and ANN, on Mexico dataset to predict COVID-19 infection. They obtained the highest (94.99%) prediction accuracy with decision tree, maximum (93.34%) sensitivity with SVM and maximum (94%) specificity with NB. Zeroual et al. [22] compared five deep learning models, recurrent neural network, long short-term memory, bidirectional LSTM, gated recurrent units, and variational autoencoder algorithms, to predict COVID-19 prognosis in Italy, Spain, France, China, USA, and Australia and reported superior performance of variational autoencoder as compared to others. Zoabi et al. [23] established a machine learning approach trained on the data of 51,831 individuals of the Israeli Ministry of Health. The model predicted high accuracy with eight binary features like sex, age ≥ 60, known contact with infected individuals, and the initial five (cough, fever, sore throat, dyspnoea, and headache) clinical symptoms. Aljameel et al. [24] reported a prediction model for early identification of COVID-19 by using 287 samples collected from the King Fahad University Hospital, Saudi Arabia. They analysed the data with three classified algorithms, random forest, logistics regression, and extreme gradient boosting.

## 2. Materials and Methods

### 2.1. Proposed System

The IoT is a proposed system where everything is connected to the Internet. It bridges the gap between the man and the machine. Using emerging technology, IoT has impacted numerous fields of human endeavours greatly including the healthcare system. It could change the existing healthcare system merely by using advanced sensors and cloud computing platform. IoT, an advanced automation system that uses big data concept, makes it possible to connect every asset through the web and helps design a smart healthcare system. As IoT handles big data, it is hard for the healthcare professionals to handle and manage it. Thus, the medical professionals require chronicled data to predict a disease. Although various kinds of machine learning algorithms have been used since long to predict a disease, the biggest challenge in the machine learning algorithm is to tune the various parameters. Proper tuning of the parameters results in efficient prognosis and diagnosis of a disease.

### 2.2. Significance of the Proposed System

The present work proposes a framework of e-healthcare system by using artificial intelligence, machine learning, and statistics for disease prognosis. In the proposed system, the patient's data are collected stored in cloud by using IoT sensors and transmitted to the web server (mobile app) through the IoT agent. The cloud shares the data over social insurance frameworks, and various machine learning algorithms are executed to process the data. The response is sent to healthcare professionals to monitor and suggest proper actions. The block diagram of the proposed system is shown in Scheme 1.

In this proposed model, six data prediction techniques are used and their performances are compared to provide better and reliable quality service for the healthcare system. Data prediction techniques used are k-nearest neighbor, support vector machines, decision tree, random forest, gradient boosting classifier, Naïve Bayes, and logistics regression.

### 2.3. Proposed Methodology

The main objective of this work was to forecast the probability of a patient suffering from COVID-19 infection using computer-aided diagnosis/prognosis system. To deliver this work, different ML techniques were implemented on the given dataset which is analysed and described in this study. Application of machine learning to predict COVID-19 infection provides a new and more reliable direction to the healthcare professionals for an early-stage disease diagnosis. It helps researchers predict the rising COVID-19 cases at the symptom stage and also helps in preventing the disease by taking due diligent precautions.

### 2.4. Data Source

The dataset used for the work was accessed from Kaggle site [25]. The dataset could be collected in a CSV file and uploaded in a Jupiter notebook for analysis with the Python software. The dataset contained a total of 5434 data samples and 19 features/parameters related to the patient symptoms as detailed in Table 1. Seven machine learning algorithms were implemented in this work for COVID-19 prognosis with maximum possible accuracy and create an automated system for COVID-19 detection.

### 2.5. Data Preprocessing

The dataset contained vast numbers of null values and outliers which might affect the accuracy of the model. To remove these noisy data, the datasets were preprocessed and the null values were removed to help increase the efficacy of the models. After cleaning the dataset, the data were transformed to a new form by using the process of smoothing and normalisation. The dataset was classified into testing and training set which was implemented on several machine learning models to compare the accuracy score. The various machine learning algorithms used in this research are discussed below.

#### 2.5.1. Logistics Regression

This classifier, used for classification and data analysis, is based on supervised algorithm. It is a type of regression model when data modeling requires sigmoid function [26].

(1) $$\begin{array}{c} \text{Sigmoid function},g\left(y\right)=\frac{1}{1+e^{-y}}. \end{array}$$

Here, the regression model is built to predict the probability and measure the learning rate; thus, it is also considered as a probabilistic classifier. As it is based on classification technique, the output or target variables take only the discrete values for features/parameters as input values.

#### 2.5.2. Support Vector Machines (SVM)

This classifier, used for both classification and regression analysis, is based on supervised algorithm. This classifier is a margin-based classifier as it differentiates the data between margin and hyperplane and distinctly classifies the dataset into classes.

It has the capability to work on text classification problem. It deals with two group classification problems by giving the model sets for labeled type of training data for each category. The hard margin type of support vector model optimisation problem can be solved by using the Lagrange multiplier method.

#### 2.5.3. Random Forest (RF) Model

This classifier is the ensemble learning classifier. It is used for both classification and regression analysis. It consists of a set of trees in which each tree is capable of providing a set of predictor values [27]. Overall, the decision trees are weak classifier and they are merged to form a random forest model. Random forest model does not have cross-validation, while the other classifiers like decision tree and k-NN model have cross-validation. In this classifier, a greater number of trees result in more accuracy. Random forest classifier logic uses entropy, gain ratio, and Gini index.

(2) $$\begin{array}{c} \text{Entropy }\left(N\right)=-\overset{n}{\underset{i=1}{\sum }}\pi \;\log_{2}\pi ,\\ \text{Gini }\left(N\right)=1-\overset{M}{\underset{I=1}{\sum }}\pi^{2},\\ {\text{Gini}}_{A}\left(N\right)=\frac{N_{1}}{N}\text{Gini}\left(N_{1}\right)+\frac{N_{2}}{N}\text{Gini}\left(N_{2}\right). \end{array}$$

#### 2.5.4. Decision Tree (DT) Model

This classifier is based on classification algorithm while it works on numerical and categorical data. It is required to create tree-shaped graph while analysing the data. The analysis of decision trees is based on three nodes (root node, interior node, and leaf node). The idea behind such decision algorithm includes the best attributes using information gain and the gain ratio. It makes a decision tree based on that attribute and breaks into subdatasets. Further, it starts building the tree and process repetition recursively.

(3) $$\begin{array}{c} \text{Information }\left(M\right)=-\overset{n}{\underset{i=1}{\sum }}\pi \;\log_{2}\pi ,\\ {\text{Information}}_{A}\;\left(M\right)=\overset{m}{\underset{j=1}{\sum }}\frac{M_{J}}{M}\;X\text{ Information }\left(M_{j}\right),\\ {\text{Split}}_{A}\;\left(M\right)=-\overset{m}{\underset{j=1}{\sum }}\frac{M_{J}}{M}\;\log_{2}\frac{M_{J}}{M},\\ \text{Gain Ratio }\left(N\right)=\frac{\text{Gain }\left(N\right)}{{\text{Split}}_{A}\;\left(M\right)}. \end{array}$$

#### 2.5.5. k-Nearest Neighbor (k-NN)

Based on supervised algorithm, k-nearest neighbour technique is based on the nearest neighbour data points concept. By using different distance metric concept, the nearest neighbour data point could be deciphered. Although inefficient for large dimensional dataset, k-NN technique is easy to implement. It is a nonparametric model used to solve classification and regression problems. The object is classified depending on the nearest neighbour using the classification technique. The calculation of the nearest neighbor is measured using the Euclidean distance.

(4) $$\begin{array}{c} \text{Euclidean Distance},\;d{\left(a,b\right)}^{2}={\left(b_{1}-a_{1}\right)}^{2}+{\left(b_{2}-a_{2}\right)}^{2}. \end{array}$$

Here, the input consists of the closest or nearest neighbour in the dataset to deploy the model. The classifier assumes similar attributes existing in closer proximity. After loading the data and choosing the nearest neighbour, the distance between query and original example is calculated and the numbers of entries are sorted in the collection [28].

#### 2.5.6. Naïve Bayes (NB)

This classifier is based on supervised algorithm. A classification technique by Baye's theorem, it finds out the probability of attributes not having any correlation with each other. All attributes contribute independently to the probability. The probability could be calculated by building the frequency table and likelihood table. Further, the test phase from the likelihood table needs to be found out after the training is done. The Baye's theorem equation is

(5) $$\begin{array}{c} P\;\left(B/A\right)=\frac{P\left(B/A\right).P\left(B\right)}{P\left(A\right)}, \end{array}$$

where *P*(*B*/*A*) is the posterior probability, *P*(*B*) is the class prior probability, *P*(*A*) is the predictor prior probability, and *P*(*A*/*B*) is the predictor probability.

#### 2.5.7. Gradient Boosting Machine (GBM)

This classifier is the most popular among all the boosting algorithms where each predictor corrects its preceding predictor's error. Each predictor in the model is trained well using the errors of the preceding predictors. The base learner in the machine is the classification and regression trees [29]. The major parameter used in this technique is the shrinkage which refers to the prediction of each tree when the model is shrunk after multiplying the learning rate that ranges between 0 and 1. Since all trees are trained, the final prediction is done by the following formula:

(6) $$\begin{array}{c} x\left(\text{pred}\right)=x1+\left(\eta *r1\right)+\left(\eta *r2\right)+\cdots \cdots .+\left(\eta *rn\right). \end{array}$$

The algorithm is used to classify gradient boosting classifier, and the class is called the gradient boosting regressor (GBR).

## 3. Results

Count plot shows that 4383 patients suffered from COVID-19 and 1051 patients did not (Figure 1). Pie plot shows that 80.7% patients had COVID-19 infection and 19.3% did not have (Figure 2).

3620 patients had breathing problem and 1814 did not out of 5434 data samples. Similarly, 4273 patients suffered from fever and 1161 did not, 4307 patients had dry cough and 1127 did not, 3953 patients had sore throat and 1481 did not, and 2952 patients had running nose and 2482 did not (Figure 3).

Also, 2514 patients had asthma tendency and 2920 did not, 2565 patients had chronic lung disease and 2869 did not, 2736 patients had headache and 2698 did not, 2523 patients had heart disease and 2911 did not have, and 2588 patients suffered from diabetes and 2846 did not. Patients with heart disease, diabetes, headache, asthma, hypertension, fatigue, gastrointestinal issue, and prior contact with COVID-19 patient had more probability of suffering from COVID-19 infection than those that followed COVID appropriate measures (such as wearing a mask and sanitising regularly) and had no associated health or sociological issues.

Pearson, Spearman, and Kendallau correlation coefficient are presented in Table 2. Features like wearing a mask and sanitisation from market are not considered as they contained null values. As running nose, chronic lung and heart diseases, gastrointestinal issues are strongly correlated, these features are removed. The correlation matrix after these data cleaning is shown in Figure 4.

### 3.1. Confusion Matrix

This table is considered to visualise the classification of classification model. It contains positive, negative observation of actual class and positive, negative observation of predicted class. The four observations are TP1 (true positive), FN1 (false negative), TN1 (true negative), and FP1 (false positive). The confusion matrix and the performance measurement parameters of k-NN models are presented in Figure 5 and Table 3.

This curve is used to evaluate binary classification and plots true positive observations by the false positive observations. AUC is used to measure the performance by distinguishing the positive and negative observations.

The area under the curve value obtained for k-NN algorithm was found to be 0.98 (Figure 6). It represents that k-NN model was able to reliably prognose COVID-19 infection up to 98%. k-NN model performance measure matrices are presented in Table 4 and are used to calculate sensitivity, specificity, precision, and accuracy.

#### 3.1.1. Sensitivity (Recall)

This is used to calculate the true positive prediction by the total number of positive prediction. Recall represents correctly predicted positive class. The best sensitivity rate is 1.0 and the worst rate is 0.

(7) $$\begin{array}{c} \text{Sensitivity}=\frac{\text{TP}1}{\text{TP}1+\text{FN}1}. \end{array}$$

#### 3.1.2. Specificity

This is used to calculate true negative predictions by the total number of negative prediction. The best specificity rate is 1.0 and the worst rate is 0.

(8) $$\begin{array}{c} \text{Specificity}=\frac{\text{TN}1}{\text{TN}1+\text{FP}1}. \end{array}$$

#### 3.1.3. Precision

It represents the actual number of positive class from total number of positive classes.

(9) $$\begin{array}{c} \text{Precision}=\frac{\text{TP}1}{\text{TP}1+\text{FP}1}. \end{array}$$

#### 3.1.4. Accuracy

It is used to calculate the true observations to the total number of observations. True observations are TP and TN.

(10) $$\begin{array}{c} \text{Accuracy}=\frac{\text{TP}1+\text{TN}1}{\text{TP}1+\text{TN}1+\text{FP}1+\text{FN}1}. \end{array}$$

#### 3.1.5. F1-Score

It is the harmonic mean between precision and sensitivity.

(11) $$\begin{array}{c} FI=\frac{\left(1+\beta^{2}\right)\text{Precision}.\text{Sensitivity}}{\beta^{2}\left(\text{Precision}+\text{Sensitivity}\right)}, \end{array}$$

where *β* is a constant which is commonly 1, 2, or 0.5.

(12) $$\begin{array}{c} F1=\frac{\text{TP}1.\text{TP}1}{\text{TP}1+\text{TP}1+\text{FP}1+\text{FN}1},\\ FI=\frac{2.\text{TP}1}{2.\text{TP}1+\text{FP}1+\text{FN}1}. \end{array}$$

## 4. Discussion

This piece of research work detects (prognoses) whether or not a patient is likely to suffer from COVID-19 infection by observing the patients' symptoms. This research was done on machine learning classification techniques using Naïve Bayes, decision tree, random forest, k-nearest neighbor, support vector machine, logistics regression, and gradient booster. The dataset was collected from Kaggle site and processed using python open access software in Jupyter notebook. The data was analysed and split into a training set and a test set. Different ML models are implemented on the dataset, and the performance of each of the model is described in terms of accuracy. Performance report of the various test models executed in the study is given in Table 5. The percentage of accuracy score is presented in Table 6, and the accuracy comparison of each of the model are depicted in Figure 7. From the accuracy plot, it was concluded that k-NN was more accurate (97.97%) followed by decision tree (97.79), support vector machine (97.42), logistics regression (96.50), random forest (90.66), gradient boosting classifier (87.77), and Naïve Bayes (73.50) in COVID-19 prognosis based on the given dataset and the defined features/parameters.

Out of all the models compared for reliability, k-NN model was found to be the best. It was found that k-NN model with a prediction accuracy of 98% performed better as compared to other six algorithms. We have also compared the results of our study with some other reported models (Table 7), which suggests that our models are effective and give better results [30–34]. We have used a 10-fold cross-validation method for improving the performances of our models. In future, this research may help healthcare professionals to predict and diagnose COVID-19 at an early stage. This would be useful especially for the patients in remote locations with low access to immediate medical facility. COVID-19 prognosis could also be done using other machine learning and deep learning approaches with potentially better accuracy. This study is bound to provide ample references for further development in this field at a global scale. However, more robust datasets as inputs are strongly recommended to achieve this.

## 5. Conclusion

Many countries including India are still struggling to fight against this deadly corona pandemic as the cases are rising daily. Each day comes as a new challenge with ever larger quantity of COVID-19 cases and data. To address this, research to develop medicines to treat and vaccines to prevent COVID-19 is being pursued at global scale. This paper compares seven machine learning algorithms in terms of their accuracy in COVID-19 prognosis; machine learning algorithms are implemented to predict/prognose COVID-19 infection in India and elsewhere. Also, the AUC and various performance measurement metrics like accuracy, precision, recall, and F1-score of k-NN model are discussed. The work provides a precursor to design an automated COVID-19 prognosis system using IoT and machine learning algorithms. The risk rate was 65-80% with the four critical symptoms (fever, dry cough, breathing issue, and sore throat) out of the 10 parameters/features considered from the 19 total possible parameters/features. So, these four critical parameters could be recommended as the strong prognosis bioindicators.

## Figures and Tables

**Scheme 1:** Proposed model for COVID-19 prognosis.

**Figure 1:** Count plot for the numerous patients suffering from COVID-19 (yes) and that did not (no).

**Figure 2:** Pie plot for the patients suffering from COVID-19.

**Figure 3:** Probability of patients suffering from COVID-19 with relevant symptoms.

**Figure 4:** Obtained correlation matrix for the given dataset after data cleaning operation.

**Figure 5:** Confusion matrix of k-NN.

**Figure 6:** AUC plot of k-NN model.

**Figure 7:** Accuracy comparison plot of different ML models.

**Table 1:** Features of the dataset.

Sl. no.	Features	Description
1.	Breathing problem	*T* = 67%; *F* = 33%
2.	Fever	*T* = 79%; *F* = 21%
3.	Sore throat	*T* = 73%; *F* = 27%
4.	Dry cough	*T* = 79%; *F* = 21%
5.	Hyper tension	*T* = 51%; *F* = 49%
6.	Abroad travel	*T* = 54.9%; *F* = 45.1%
7.	Contact with COVID patient	*T* = 50.2%; *F* = 49.8%
8.	Attended large gathering	*T* = 53.8%; *F* = 46.2%
9.	Visited public exposed places	*T* = 51.9%; *F* = 48.1%
10.	Family working in public exposed places	*T* = 58.4%; *F* = 41.6%

T: true; F: false.

**Table 2:** Different correlation coefficient of the given dataset.

Types of correlation	Pearson	Spearman	Kendallau
Highest positive correlation	0.503	0.503	0.503
Highest negative correlation	-0.016	-0.016	-0.016
Lowest correlation	0.002	0.002	0.002
Mean correlation	0.139	0.139	0.139

**Table 3:** Confusion matrix report of k-NN.

Performance parameter	Description	k-NN
TP1	Predicted and actual values are positive	862
TN1	Predicted and actual values are negative	203
FP1	Predicted value is positive but actual value is negative	2
FN1	Predicted value is negative but actual value is positive	20

**Table 4:** Classification report of k-NN model.

Performance matrix	Precision	Recall	F1-score	Support
0	0.91	0.99	0.95	205
1	1.00	0.98	0.99	882
Accuracy	—	—	0.98	1087
Macro average	0.95	0.98	0.97	1087
Weighted average	0.98	0.98	0.98	1087

**Table 5:** Performance report of the various test models executed in the study.

Algorithm	TP	TN	FP	FN	Accuracy	Sensitivity	Precision	F1-score
Logistics regression	852	208	9	18	96.50	0.97	0.98	0.98
Random forest	821	200	54	51	90.66	0.94	0.93	0.93
Decision tree	890	172	20	4	97.79	0.99	0.97	0.98
Linear SVM	885	174	17	11	97.42	0.98	0.98	0.98
Naïve Bayes	558	233	0	285	73.50	0.66	1.00	0.79
Gradient boosting classifier	814	213	55	88	87.77	0.90	0.93	0.91

**Table 6:** Accuracy score obtained by ML models.

ML models	Accuracy score	Run time (seconds)
k-NN	97.97	0.543
Decision tree	97.79	0.024
Support vector machines	97.42	0.217
Logistics regression	96.50	0.053
Random forest	90.66	5.423
Gradient boosting classifier	87.77	0.523
Naïve Bayes	73.50	0.013

**Table 7:** Performance comparison of proposed work with other reported works.

	Model for prediction	Accuracy	Specificity	Sensitivity	AUC
Brinati et al. [30]	Random forest	82	—	—	84
Tschoellitsch et al. [31]	Random forest	81	—	—	74
Tordjman et al. [32]	Logistics regression	—		80.3	88.9
Soltan et al. [33]	Extreme gradient boosting tree	—	94.8	77.4	99
Alakus and Turkoglu [34]	LSTM	86.66	—	99.42	62.50
Proposed work	k-NN	97.97	0.98	0.98	98
	Random forest	90.66	0.94	0.93	98
	Logistics regression	96.50	0.97	0.98	93
	SVM	97.42	0.98	0.98	89
	Decision tree	97.79	0.99	0.97	95
	Gradient boosting classifier	87.77	0.90	0.93	97

## Data Availability

The data used to support the findings of this study are available from the corresponding author upon request.
